The article "Comparison of the Effects of Carperitide and Tolvaptan on Patients with Left Ventricular Dysfunction: A Two-Center Retrospective Study" was published in 2017. Journal: Cardiol Res Pract.

# Comparison of the Effects of Carperitide and Tolvaptan on Patients with Left Ventricular Dysfunction: A Two-Center Retrospective Study

**DOI:** 10.1155/2017/6935342

**Published:** 2017-07-12

**Authors:** Chikahiko Koeda, Shohei Yamaya, Maiko Hozawa, Masayuki Sato, Kazuhiro Nasu, Tomohiro Takahashi, Katsutoshi Terui

**Affiliations:** ^1^Division of Cardioangiology, Department of Internal Medicine, Iwate Medical University, Iwate, Japan; ^2^Department of Cardiology, Iwate Prefectural Kuji Hospital, Iwate, Japan; ^3^Department of Emergency, Iwate Medical University, Iwate, Japan

## Abstract

In patients with left ventricular (LV) dysfunction, diuretics can reduce blood pressure and lead to electrolyte abnormalities. The aim of this study was to compare the effects of tolvaptan (T group) and carperitide (C group) in these patients. Sixty-one consecutive patients admitted to the Iwate Prefectural Kuji Hospital or the Emergency Center of the Iwate Medical University between July 2011 and April 2015 were included in this study. These patients had acute heart failure (HF) and were initially treated with furosemide. Patients were excluded from the study if they received combined carperitide and tolvaptan, if they received tolvaptan or cardiotonic drugs prior to the study period, if their LV ejection fraction was ≥40%, and if they had renal dysfunction (serum creatinine > 2.0 mg/dL). There were no differences in the change in serum electrolytes in both groups, and none of the patients in the T group received supplementary dobutamine therapy. Oxygen administration was stopped successfully after a significantly shorter treatment period in the T group. These findings suggest that patients treated with tolvaptan did not require dobutamine as frequently as those treated with carperitide and indicated that tolvaptan may improve respiratory function more rapidly in patients with LV dysfunction.

## 1. Introduction

Diuretic drugs, including loop diuretics and natriuretic peptides, are used frequently as a conventional therapy in patients with acute heart failure (HF). Carperitide is a B-type natriuretic peptide that can produce therapeutic benefits because it has a diuretic effect and a vasodilator action and inhibits activation of the renin aldosterone system [1]. It is an important therapeutic agent for HF and is currently used in 69.4% of these cases in Japan [2]. However, older patients and those with a left ventricular (LV) ejection fraction of <35% may show reduced blood pressure (BP) after carperitide administration [3], and those with LV dysfunction were more likely to be nonresponders in the COMPASS study of carperitide [4]. In a study of nesiritide, another B-type natriuretic peptide, approximately 80% of the participants had LV dysfunction and many showed dose-dependent decreases in BP, with no confirmed improvements in prognostic predictors [5]. Although B-type natriuretic peptides have significant therapeutic benefits, these agents do not currently provide sufficient effects in patients with LV dysfunction. Loop diuretic drugs activate neurohormonal factors, reduce BP, and reduce serum osmotic pressure. The associated hyponatremia limits their use in patients with HF because hyponatremia is recognized as an independent predictor of poor prognosis in patients with LV dysfunction [6]. Hyponatremia was reported in 33.7% of patients with an initial LV ejection fraction of <35% [7]. Thus many patients with LV dysfunction may show resistance to conventional carperitide therapy, which might negatively affect the results of the mega clinical trial.

Patients with LV dysfunction and hyponatremia showed increased levels of vasopressin, which has two functions, to constrict BP and to keep fluid in body, and decreases LV output. Many cases of congestion symptoms and electrolyte abnormalities due to fluid retention have been reported [8, 9]. Tolvaptan is a vasopressin receptor antagonist which affects hemodynamics favorably; recent studies have investigated its clinical efficacy in these patients [10, 11].

The aim of the present study was to evaluate the effects of tolvaptan on LV dysfunction retrospectively by comparing the clinical features of carperitide-treated patients (C group) with those of tolvaptan-treated patients (T group).

## 2. Materials and Methods

### 2.1. Patients

Sixty-one consecutive patients (37 male and 24 female patients) were enrolled in this retrospective study. These patients were admitted to the Iwate Prefectural Kuji Hospital or the Critical Care and Emergency Center of Iwate Medical University Hospital between July 2011 and April 2015 with acute HF and were initially treated with loop diuretics. Patients were excluded from the study if they had received combination therapy with carperitide and tolvaptan or if they had been treated with tolvaptan or cardiotonic drugs in an outpatient setting. They were also excluded if their LV ejection fraction was ≥40% or they showed signs of renal failure (serum creatinine > 2.0 mg/dL) on admission. In addition, there were no patients who underwent intubation and mechanical respiratory support.

### 2.2. Study Design and Data Collection

A retrospective cohort design was employed on the basis of a medical chart review. The following data were obtained at the time of admission and within 24 hours after drug administration: sex, age, anthropometric measures, New York Heart Association (NYHA) class, medical history, comorbidities, vital signs, laboratory data, echocardiographic findings, electrocardiogram, urine and intake volume, hospitalization, mortality, the number of days before beginning the combination of loop diuretic and target drug (carperitide or tolvaptan), use of cardiotonic drugs, and changes in serum electrolytes or vital signs. Furthermore, we investigated the number of days between beginning the test therapy and stopping oxygen administration because this can provide an objective measure of respiratory function.

### 2.3. Statistics

We compared clinical measures in the C and T groups on admission and after test drug administration. Statistical comparisons between the C and T groups were made using the unpaired *t*-test (parametric data) or Mann–Whitney *U*-test (nonparametric data). Categorical variables were analyzed using the chi-square test. All analyses were performed using the SPSS software package (Chicago, IL, USA), and a *p* value of <0.05 was considered to be statistically significant.

## 3. Results and Discussion

### 3.1. Results

#### 3.1.1. Baseline Patient Characteristics

Table 1 shows the patient data prior to administration of carperitide or tolvaptan. The mean age of the C group (*n* = 46) was 6 years older than that of the T group (*n* = 15), although this difference was not statistically significant (*p* = 0.15). There were more males than females in both study groups. The mean body mass index of the T group was slightly higher than that of the C group (*p* = 0.05). The NYHA class was ≥III in all cases and there was no difference in the furosemide dose administered prior to carperitide or tolvaptan.

#### 3.1.2. Medical History

There were no differences in the past histories of HF, hypertension, diabetes mellitus, brain infarction, or medication histories relating to angiotensin converting enzyme inhibitors, angiotensin II receptor blockers, antialdosterone compounds, or *β*-blockers. The patients with hyperlipidemia were higher in the T group (*p* = 0.05). The causes of HF in these patients are shown in Table 1; in patients where no definitive diagnosis was available (“Others”), hypertensive heart disease, takotsubo cardiomyopathy, and arrhythmia were suspected.

#### 3.1.3. Vital Signs and Laboratory Data on Admission

As shown in Table 1, there were no differences in the systolic and diastolic BPs or heart rates of the study groups. The serum sodium level was slightly lower in the C group than in the T group (*p* = 0.02), while there were no significant group differences in the blood urea nitrogen or serum creatinine levels. Sinus rhythm on electrocardiogram was noted in 20 cases (43%) in group C and 8 cases (53%) in group T. There were no differences in LV ejection fraction between the two groups, but the LV end‐diastolic dimension and the estimated LV volume were significantly higher in the T group than in the C group (*p* < 0.05 for both analyses). There were no significant group differences in the estimated stroke volumes or right ventricular pressures.

#### 3.1.4. Vital Signs and Laboratory Data upon Initiation of Carperitide or Tolvaptan Administration

As shown in Table 2, there was a significantly shorter delay before therapy initiation in the C group than in the T group (*p* < 0.001). Immediately prior to therapy initiation, systolic and diastolic BPs were significantly lower in the T group than in the C group (*p* < 0.05 for both comparisons). The serum sodium level was significantly lower in the C group, as compared with the T group (*p* = 0.03).

After the initiation of carperitide or tolvaptan therapy, there were no significant differences in the durations of hospitalization or therapy administration in the C and T groups. The 5 fatalities all occurred in the C group (11%). There were no significant differences in the furosemide dose administered to the two study groups. In addition, the 28 cases in which dobutamine was used after a mean of 2.1 ± 5.4 days were all in the C group (61%). The time before successfully stopping oxygen administration was 20% shorter in the T group than in the C group (*p* = 0.04). There were no significant group differences in the change in renal function and the serum electrolytes. The C group showed a significantly greater decrease in systolic BP than the T group (*p* < 0.001), and the change in diastolic BP was also smaller in the T group than in the C group (*p* = 0.001). Although the mean urine volume in the 3 days after drug initiation was greater in the T group than in the C group, this difference was not statistically significant because the mean intake volume was unclear.

### 3.2. Discussion

This retrospective study of HF patients with an EF of <40% found that 61% of the C group received additional dobutamine within two days of carperitide therapy initiation, while those in the T group did not require dobutamine. There were no intergroup differences in the doses of furosemide and combination treatment in the two groups. Thus, the findings are comparable to those of studies comparing tolvaptan monotherapy and combination therapy with carperitide and dobutamine. The present study found no differences in serum electrolyte levels or renal function in the T and C groups. The time between therapy initiation and successful cessation of oxygen administration was significantly shorter in the T group than in the C group and none of the patients in the T group died during the study period, even though their heart expansion progressed. In contrast, 5 of the patients in the C group died during the study. These results suggested that the therapeutic effects of monotherapy with tolvaptan may not be inferior to those of combined carperitide and dobutamine treatment in patients with LV dysfunction. The release of vasopressin positively correlated with HF stage [12], and the demand of tolvaptan may rise as HF stage progresses. Even though tolvaptan was not shown to produce prognostic improvements in a large-scale clinical trial [13], this compound may provide an effective treatment strategy for the subgroup of patients with LV dysfunction for the following reasons. First, it has been reported that aquaporin-defined responders may have a better prognosis with tolvaptan [14].

Second, although cardiac index remained unchanged, the pulmonary vascular resistance index decreased after tolvaptan treatment [15]. Finally, the result in this study indicated that tolvaptan use can reduce cardiotonic dose which is cause of the poor-prognosis factor.

Although 61% of the C group was treated with dobutamine, systolic BP showed a large decrease after carperitide infusion. In contrast, no significant change in BP was observed in the T group. The results of this study are consistent with those of a previous investigation of tolvaptan in patients with HF and reduced LV ejection fraction < 50% or systolic BP < 140 mmHg, who showed a greater effect of diuretics on BP than did patients with HF and a preserved ejection fraction [16]. However, these results may be influenced by the difference in the time delay prior to starting carperitide or tolvaptan therapy. The T group received only furosemide for approximately 3 days after hospitalization, allowing their stroke volumes and BP to decrease without dobutamine administration. On the other hand, the majority of the C group received carperitide on admission and yet 61% of these patients subsequently required dobutamine. There was a clear difference in group BPs at the time of treatment initiation, whereby the T group showed a significantly lower systolic BP than did the C group. Accordingly, this bias made it difficult to evaluate the effect of tolvaptan on BP.

There were limitations to this study related to the small number of cases and the retrospective analysis, although we aimed to minimize bias by using strict exclusion criteria. Bias affected normality in the baseline features of the study groups and this was difficult to correct for, even with an analysis of covariance. Furthermore, we wanted to reconsider our findings according to the various types of acute HF and compare tolvaptan responders and nonresponders; however, these were not possible due to the sample size. The larger number of patients in the C group indicated a tendency for clinicians to prescribe the more established therapy. These findings reflected the real-world use of tolvaptan, as a new drug.

## 4. Conclusions

The findings of this study indicated that tolvaptan use was associated with lower rates of dobutamine administration, as compared with carperitide, and that tolvaptan may improve respiratory function in patients with LV dysfunction. This indication that tolvaptan treatment may not be inferior to carperitide treatment in patients with LV dysfunction suggested that further examination of this was warranted in a future prospective study.

## Figures and Tables

**Table 1:** Baseline characteristics. The values are expressed in mean (standard deviation) and median (interquartile range). NYHA = New York Heart Association; ACE = angiotensin converting enzyme; ARB = angiotensin II receptor blocker; LV = left ventricular.

	Carperitide	*n*	Tolvaptan	*n*	*p* value
Age (year)	82 (77–88)	46	74 (62–88)	15	0.15
Sex (male)	28 (61%)	46	9 (60%)	15	1
Body mass index (kg/m^2^)	22.1 ± 3.9	40	24.8 ± 5.2	15	0.05
NYHA class					
III	7 (15%)	46	2 (13%)	15	1
IV	39 (85%)	46	13 (87%)	15	1
Furosemide dose (mg)	20 (0–40)	46	20 (0–40)	15	0.77
Previous therapies					
ACE inhibitors	9 (20%)	46	2 (13%)	15	0.72
ARBs	9 (20%)	46	5 (27%)	15	0.3
Aldosterone blockers	9 (20%)	46	2 (13%)	15	0.72
*β*-Blockers	15 (33%)	46	4 (27%)	15	0.76
Medical history					
Heart failure	31 (67%)	46	9 (60%)	15	0.76
Hypertension	26 ( 57%)	46	4 (27%)	15	0.07
Diabetes mellitus	8 (17%)	46	1 (7%)	15	0.43
Hyperlipidemia	2 (4%)	46	4 (27%)	15	0.05
Brain infarction	17 ( 37%)	46	2 (13%)	15	0.12
Type of heart failure					
Diastole cardiomyopathy	18 (39%)	46	3 (20%)	15	0.22
Ischemic heart disease	19 (41%)	46	3 (20%)	15	0.22
Hypertrophic cardiomyopathy	1 (2%)	46	0	15	1
Others	8 (17%)	46	9 (60%)	15	0.03
On admission					
Systolic blood pressure (mmHg)	144.3 ± 26.1	46	140.3 ± 22.4	15	0.59
Diastolic blood pressure (mmHg)	89.3 ± 14.5	46	93.1 ± 18.1	15	0.42
Heart rate (bpm)	100 (90–109)	46	101 (83–122)	15	0.67
Serum sodium (mEq/L)	139.9 ± 3.4	46	142.3 ± 2.9	15	0.02
Serum potassium (mEq/L)	4.3 ± 0.5	46	4.1 ± 0.3	15	0.56
Blood urea nitrogen (mg/dL)	28.2 ± 10.6	45	23.8 ± 8.7	15	0.16
Serum creatinine (mg/dL)	1.2 ± 0.4	46	1.0 ± 0.4	15	0.16
On initiation of therapy					
Systolic blood pressure (mmHg)	142.4 ± 24.6	46	121.9 ± 18.1	15	0.004
Diastolic blood pressure (mmHg)	88.7 ± 15.2	46	78.0 ± 13.2	15	0.02
Heart rate (bpm)	98 (90–105)	46	98 (84–119)	15	0.73
Serum sodium (mEq/L)	140.2 ± 3.7	46	142.5 ± 2.6	15	0.03
Serum potassium (mEq/L)	4.3 (4.2–4.3)	46	4.0 (3.9–4.2)	15	0.04
Blood urea nitrogen (mg/dL)	27.1 (19.2–38.0)	45	23.5 (19.1–31.0)	15	0.18
Serum creatinine (mg/dL)	1.2 ± 0.4	46	1.0 ± 0.3	15	0.12
Urine before combination therapy (mL)	1070 (650–1153)	5	1266 (858–1750)	7	0.29
Electrocardiogram					
Sinus rhythm	20 (43%)	46	8 (53%)	15	0.56
Echocardiography					
End‐diastolic dimension (mm)	51.7 ± 9.8	42	56.7 ± 7.3	15	0.04
LV ejection fraction (%)	29.1 ± 7.3	46	26.9 ± 8.3	15	0.22
Diastolic LV volume (mL)	131.7 ± 42.5	17	183.3 ± 48.9	11	0.001
Systolic LV volume (mL)	93.4 ± 31.5	17	139.3 ± 40.7	11	0.001
Stroke volume (mL)	35.6 (20.7–48.8)	17	41.1 (28.7–51.0)	11	0.32
Right ventricle pressure (mmHg)	48.4 ± 11.5	40	49.6 ± 8.2	13	0.72

**Table 2:** After the initiation of carperitide or tolvaptan therapy. The values are expressed in mean (standard deviation) and median (interquartile range).

	Carperitide	*n*	Tolvaptan	*n*	*p* value
Hospitalization (day)	31 (20–43)	46	30 (21–34)	15	0.93
Duration of combination therapy (day)	9.0 ± 5.8	45	9.3 ± 5.6	14	0.87
Fatalities	5 (11%)	46	0	15	0.32
Combined furosemide dose	40 (20–60)	46	40 (20–60)	15	0.76
Time before combination therapy initiation	0.5 ± 1.3	46	2.9 ± 3.4	15	<0.001
Received dobutamine	28 (61%)	46	0	15	<0.001
After combination therapy initiation					
Time taken to stop oxygen administration (day)	11 (7–17)	38	9 (4–10)	14	0.04
Systolic blood pressure (mmHg)	118.7 ± 21.6	46	121.6 ± 17.7	15	0.64
Diastolic blood pressure (mmHg)	69 (62–77)	46	72 (62–81)	15	0.54
Heart rate (bpm)	88 (78–97)	46	86 (68–100)	15	0.9
Serum sodium (mEq/L)	142.6 ± 3.6	46	143.5 ± 2.8	15	0.4
Serum potassium (mEq/L)	3.9 ± 0.5	46	4.0 ± 0.4	15	0.63
Blood urea nitrogen (mg/dL)	23.1 (18.8–31.9)	46	22.1 (19.1–25.3)	15	0.44
Serum creatinine (mg/dL)	1.2 ± 0.4	46	1.0 ± 0.3	15	0.1
ΔSystolic blood pressure (mmHg)	−23.7 ± 17.2	46	−0.3 ± 12.8	15	<0.0001
ΔDiastolic blood pressure (mmHg)	16.0 (10.0–27.0)	46	3.0 (−2.0–11.0)	15	0.001
ΔHeart rate (bpm)	−10.7 ± 14.2	46	−7.1 ± 18.5	15	0.43
ΔSerum sodium (mEq/L)	2.5 ± 4.1	46	1.0 ± 4.0	15	0.21
ΔSerum potassium (mEq/L)	−0.3 ± 0.5	46	0 ± 0.5	15	0.09
ΔBlood urea nitrogen (mg/dL)	−3.9 ± 9.0	45	−1.5 ± 8.4	15	0.38
ΔSerum creatinine (mg/dL)	0 ± 0.3	46	0 ± 0.2	15	0.92
Urine volume (mean of 3 days) (mL)	1418 (1019–1813)	46	1833 (1183–4833)	11	0.03
